The article "Effects of Family Participatory Nursing on Clinical Outcomes of Premature Infants in NICU and Families' Psychological Status" was published in 2022. Journal: Contrast Media Mol Imaging.

# Effects of Family Participatory Nursing on Clinical Outcomes of Premature Infants in NICU and Families' Psychological Status

**DOI:** 10.1155/2022/7420909

**Published:** 2022-07-05

**Authors:** Min Liu, Yanting Xu, Yahong Li

**Affiliations:** ^1^Teaching and Research Section of Women and Children, Quanzhou Medical College, Quanzhou, China; ^2^Department of Pediatrics, The People's Hospital Affiliated to Quanzhou Medical College, Quanzhou, China

## Abstract

The purpose of this study was to explore the effects of family participatory nursing on the clinical outcomes of premature infants in the neonatal intensive care unit (NICU) and their families' psychological status. Total of 150 premature infants were admitted to the NICU of our hospital from December 2019 to December 2021, and their families were selected by convenience sampling method and divided into control group (*n* = 78, from December 2019 to December 2020) and observation group (*n* = 72, from January 2020 to December 2021) according to the admission time. The infants in the control group were given routine nursing, while those in the observation group received family participatory nursing. In the observation group, the length of stay and duration of oxygen therapy were shorter, the weight gain speed was higher, and the incidence rate of nosocomial infection was lower than those in control groups (*P* < 0.05). The time of reaching full gastrointestinal feeding was earlier, the daily milk intake and exclusive breastfeeding rate were higher, and the feeding intolerance rate was lower in observation group than those in control group (*P* < 0.05). Observation group exhibited significantly higher body weight, Z-value of body weight, NBNA score at 7 d after hospitalization, 15-month mental development index (MDI), and psychomotor development index (PDI) scores than control group (*P* < 0.05). In addition, the families' somatization, depression and anxiety factor scores, and total score of SCL-90 in the observation group were lower than those in the control group, while each dimension score and total score of MPOC-20 were higher than those in control groups (*P* < 0.05). Family participatory nursing is of great significance in ameliorating the clinical outcomes of premature infants in the NICU, which can shorten the length of stay, improve feeding conditions, facilitate infant growth and development, and enhance their families' psychological status and nursing satisfaction.

## 1. Introduction

Due to low body weight and immature development of organs, premature infants are prone to serious health problems, so long-term monitoring in the neonatal intensive care unit (NICU) is often required [1, 2]. The NICU in China is mainly managed in a closed mode, and most families of NICU children can only visit at certain times, which is not conducive to the neurological development of the child and may affect the psychological state of the child's family to a certain extent, affecting subsequent breastfeeding and the establishment of a parent-child relationship [3, 4]. With the change in the medical humanistic concept, the closed unattended management mode of the NICU has been gradually improved in recent years. Family participatory nursing is defined as the participation of infants' families in nonmedical routine nursing of infants during hospitalization under the education and guidance of NICU specialist nurses, which can meet not only the basic physiological needs of infants but also enable families to adapt to their roles as soon as possible and improve their skills in neonatal care [5, 6]. The uncontrollable nature of preterm admission to the NICU can add to the psychological burden of families, affecting not only their own psychological well-being but also adversely affecting the systematic treatment of preterm babies [7]. At present, family participatory nursing in the NICU has been reported [8], but whether this management mode can ameliorate the psychological status of premature infants' families remains to be further studied. In this study, the effects of family participatory nursing on the clinical outcomes of premature infants in the NICU and their families' psychological status were explored, thereby providing references for clinical nursing of premature infants in the NICU.

The article "Effects of Family Participatory Nursing on Clinical Outcomes of Premature Infants in NICU and Families' Psychological Status" was published in 2022. Journal: Contrast Media Mol Imaging.

## 2. Patients and Methods

### 2.1. Patients

A total of 150 premature infants were admitted to the NICU of our hospital from December 2019 to December 2021, and their families were selected by convenience sampling method and divided into control group (*n* = 78, from December 2019 to December 2020) and observation group (*n* = 72, from January 2020 to December 2021) according to the admission time. Inclusion criteria were as follows: (1) infants with a birth weight of <2500 g and gestational age of 28–37 weeks, (2) those with a duration from birth to NICU admission for <12 hr., (3) those whose families could provide care and spend >8 hr./day with them, and (4) those whose families gave informed consent and voluntarily participated. Exclusion criteria were as follows: (1) infants receiving invasive respiratory support, (2) those complicated with congenital, hereditary, or metabolic diseases, (3) those who needed to undergo surgical treatment, and (4) those whose families had cognitive dysfunction or communication barriers. This study complied with the declaration of Helsinki. The general clinical data had no statistically significant difference between the two groups (*P* > 0.05) (Table 1).

The article "Effects of Family Participatory Nursing on Clinical Outcomes of Premature Infants in NICU and Families' Psychological Status" was published in 2022. Journal: Contrast Media Mol Imaging.

### 2.2. Methods

(1) In the control group, the infants were given routine nursing. The nurses undertook all relevant nursing tasks for the children, including basic vital sign monitoring, comfortable position adjustment, breathing management, basic nursing of the umbilicus and buttocks, touch and hearing stimulus, reasonable feeding, infection prevention, strengthening of environmental management, routine health education for families, and introduction of the infants' conditions. The infants' families could visit through the video system until the infants were discharged. The infants were followed up in the hospital every 3 months after discharge. (2) In the observation group, the infants received family participatory nursing. (1) Preparation stage: the nursing intervention team was set up, the nursing intervention system was developed, and the families received training. (a) The nursing intervention team was set up, consisting of 2 attending physicians, 1 head nurse, 2 supervisor nurses, 4 nurses, 1 prolactinist, and 1 psychological counselor. The members had different responsibilities determined according to the nature of work. Specifically, the attending physicians were responsible for disease assessment, assessment of intervention effect, answering other medical-related questions, and feasibility assessment of nursing implementation. The head nurses were mainly responsible for managing, supervising, and adjusting the nursing implementation plan. The nurses took charge of the implementation of the nursing plan. (b) The nursing intervention system was developed according to the “NICU Visiting System of Toronto Children's Center in Canada,” as follows: The nursing was given from 9:00 AM to 17:30 PM. The families' involvement should be the same ones with good health, normal cognition, basic nursing ability, and good compliance. During the nursing period, the families should be able to cooperate with the nursing intervention team, possess good awareness of cleaning and disinfection, and implement nursing under the guidance of nurses rather than acting without permission. (c) Family training: the nurses and prosthodontist provided training for the families on the admission instructions, nursing system, cleaning and disinfection, basic neonatal nursing, sensory perception intervention (touching, kangaroo mother care, and sucking care), breastfeeding, basic vital sign (body temperature, respiration, pulse, etc.) monitoring, pain manifestation and assessment, use of commonly-used instruments in the NICU, emergency handling, etc. The training could be given in the form of Microsoft Office PowerPoint (PPT) presentation, picture demonstration, one-to-one guidance, and mobile Apps. After the training, the families received assessment regarding the above training content, and they could enter the neonatal intensive care unit (NICU) for nursing after passing the assessment. (2) Implementation stage: the family participatory nursing could be started when the infants' signs became stable and no ventilator was needed, as follows: (a) the families were responsible for all the life nursing and nonmedical nursing. The father/mother of the infant entered the NICU with the nurse, and then completed bathing, diaper changing, skin care, oral care, and breastfeeding (self-provided breast milk if the father entered) under the guidance and supervision of the nurse. The families were instructed to record the general signs of the infants every day and communicate with the nurse about the infants' conditions and the daily diagnosis and treatment plan during the nursing period. (b) The families were instructed to make physical contact with the infants every day at 10:00, 12:00, 14:00, and 16:00, touch the infants' head, face, chest, abdomen, limbs, hands, feet, and back in turn in a quiet and comfortable environment, with the force from weak to strong, and rub the large muscle groups. (c) The infants' sleep cycle was introduced to the families, so as to help infants go through complete sleep cycles as far as possible and improve their sleep quality. (d) The infants' items were disinfected regularly to avoid infection, and the room temperature of the ward was kept at 28–32°C and the humidity at 60–70%. (e) Psychological support was provided for the families, and they were encouraged to actively ask questions. The questions should be patiently answered to make the families free from worry and anxiety. The families with an adverse psychological status could seek help from a psychologist. (3) Follow-up stage: the nursing ended after the infant was discharged, and the infants were followed up in the hospital every 3 months after discharge.

The article "Effects of Family Participatory Nursing on Clinical Outcomes of Premature Infants in NICU and Families' Psychological Status" was published in 2022. Journal: Contrast Media Mol Imaging.

### 2.3. Observation Indexes

(1) Hospitalization conditions: the length of stay, duration of oxygen therapy, weight growth speed, and incidence rate of nosocomial infection were recorded. Weight growth speed = (body weight at discharge - body weight at admission)/length of stay. (2) Feeding conditions: the time of reaching full gastrointestinal feeding (oral milk intake >160 mL/(kg·d)), daily milk intake, exclusive breastfeeding rate at discharge, and feeding intolerance (abdominal distension, vomiting and other symptoms, unable to digest enteral food, and gastric residue by nasal feeding >50% of the intake) rate were recorded. (3) Clinical outcomes: the body weight of infants at discharge was recorded, and its Z-value was calculated: (measured weight - mean of weight at corrected gestational age)/standard deviation of weight at corrected gestational age. At 7th day after hospitalization, the neurobehavioral function of infants was assessed using the neonatal behavioral neurological assessment (NBNA) [9]. NBNA was developed by Bao in 2003. It covers 20 items in 4 dimensions (behavioral ability, passive muscle tone, active muscle tone, primitive reflex, and general assessment) and uses a 3-level scoring method (0–40 points). The higher the score, the better the neurobehavioral function of premature infants [10–13]. The Cronbach's *α* coefficient of this scale was 0.825 in this study. Moreover, the intellectual and psychomotor development of infants at the age of 15 months was assessed using the Bayley scales of infant development (BSID). The scale developed by Nancy Bayley in 1933, which was introduced into China in 1992, includes the mental development index (MDI) and psychomotor development index (PDI), and MDI or PDI <80 points indicates developmental retardation. The Cronbach's *α* coefficient of this scale was 0.816 in this study. (4) Families' psychological status: the families' psychological status was assessed using the symptom checklist-90 (SCL-90) at discharge. Developed by derogatis in 1973, the scale was introduced into China in the 1980s, covering 90 items of 9 factors (somatization, compulsion, interpersonal relationship, depression, anxiety, hostility, phobia, paranoia, and psychosis), using a 5-level scoring method. The higher the total score, the poorer the mental health of the infants' families. The Cronbach's *α* coefficient of this scale was 0.805 in this study. (5) Nursing satisfaction: the nursing satisfaction of infants' families was assessed using the measure of processes of care 20-item (MPOC-20) at discharge. The scale was translated into Chinese by Lin et al., covering 20 items in 5 dimensions (authorization and cooperation, providing basic information, providing special information related to children, coordination and comprehensive care, and respect and supportive care) and using a 7-level scoring method. A higher total score corresponds to higher nursing satisfaction. The Cronbach's *α* coefficient of this scale was 0.821 in this study. The scales used in the text are internationally recognized and have a high degree of reliability. They are now widely used.

### 2.4. Statistical Analysis

Statistical product and service solutions (SPSS) 20.0 software (IBM, Armonk, NY, USA) was used for data analysis. Normally-distributed data were expressed as (‾*χ* ± *s*) and compared between two groups by independent-samples *t*-test. Enumeration data were expressed as [*n*(%)], and when subjected to *χ*^2^ test or Fisher's exact probability test, *P* < 0.05 was considered statistically significant.

The article "Effects of Family Participatory Nursing on Clinical Outcomes of Premature Infants in NICU and Families' Psychological Status" was published in 2022. Journal: Contrast Media Mol Imaging.

## 3. Results

### 3.1. Hospitalization Conditions in the Two Groups

In observation group, the length of stay and duration of oxygen therapy were shorter, the weight gain speed was higher, and the incidence rate of nosocomial infection was lower than those in control group (*P* < 0.05) (Table 2).

### 3.2. Feeding Conditions in the Two Groups

The time of reaching full gastrointestinal feeding was earlier, the daily milk intake and exclusive breastfeeding rate were higher, and the feeding intolerance rate was lower in observation group than those in control group, showing statistically significant differences (*P* < 0.05) (Table 3).

### 3.3. Clinical Outcomes of Infants in the Two Groups

Observation group had higher body weight at discharge, Z-value of body weight, NBNA score at 7th day after hospitalization, 15-month MDI and PDI scores than control group, and the differences were statistically significant (*P* < 0.05) (Table 4).

### 3.4. Families' Psychological Status in the Two Groups

The somatization, depression, and anxiety factor scores and total score of SCL-90 in observation group were lower than those in control group, and there were statistically significant differences (*P* < 0.05) (Table 5).

### 3.5. Nursing Satisfaction in the Two Groups

Each dimension score and total score of MPOC-20 in observation group were higher than those in control group, showing statistically significant differences (*P* < 0.05) (Table 6).

## 4. Discussion

NICU admission after birth is an important measure to improve the growth and development of premature infants. Previously [14], it was believed that the neurodevelopment of premature infants in the NICU will be adversely impacted due to early separation from their parents. Moreover, their parents are prone to mental health problems, further affecting the social and affective development of premature infants. Due to a fully closed management mode in the NICU in China, the infants' families can only visit at a specific time period and rarely have opportunities to have direct contact with infants before discharge, so the physical development of infants further becomes poor [15]. With the increasing awareness of the adverse impact of early separation of premature infants from their parents, the family-centered nursing mode has been gradually applied to the nursing intervention for premature infants in the NICU.

The article "Effects of Family Participatory Nursing on Clinical Outcomes of Premature Infants in NICU and Families' Psychological Status" was published in 2022. Journal: Contrast Media Mol Imaging.

Different from the traditional nurse-centered nursing mode, family participatory nursing promotes family participation to a new level on the basis of ability training for families. Tan et al. [16] introduced family participatory nursing to procedural pain relief for premature infants in the NICU and found that it can relieve the procedural pain of premature infants and enhance family cohesion. In this study, it was found that the hospitalization and feeding conditions in observation group were superior to those in control group. Specifically, in observation group, the length of stay and duration of oxygen therapy were shorter, the weight gain speed was higher, and the incidence rate of nosocomial infection was lower than those in control group. The time of reaching full gastrointestinal feeding was earlier, the daily milk intake and exclusive breastfeeding rate were higher, and the feeding intolerance rate was lower in observation group than those in control group. The reasons are as follows: first, the infants can eat and sleep in a quiet and comfortable environment under the family participatory nursing mode; avoiding the stimulus of lights, noises, and other personnel; and increasing the frequency of breastfeeding and daily milk intake [17]. According to a multicenter cohort randomized controlled study on breastfeeding outcomes in the NICU family participatory nursing mode [18], family participatory nursing can significantly improve the breastfeeding rate and reduce the developmental retardation of premature infants in the NICU. Second, under the family participatory nursing mode, the parents have more opportunities to have skin contact with infants, so that the infants' vital signs tend to be stable, the release of growth hormones is increased, and the infants' growth and development are facilitated [19]. In addition, the families are required to have a good awareness of cleaning and disinfection, get familiar with the matters in cleaning and disinfection of newborns' items, and disinfect these items following the requirement under the family participatory nursing mode, so the risk of nosocomial infection is reduced to a certain extent.

In terms of the clinical outcomes of infants, observation group had higher body weight at discharge, Z-value of body weight, NBNA score at 7th day after hospitalization, and 15-month MDI and PDI scores than control group, suggesting that family participatory nursing can greatly enhance the neuromotor and intellectual development of premature infants in the NICU. Premature infants often suffer from immature neurobehavioral development and have higher risks of neuromotor dysfunction and mental retardation after discharge [20]. In family education, in the core of family participatory nursing mode, the families need to improve their own nursing skills before acting as the main caregivers for premature infants in the NICU. Through PPT presentation, picture demonstration, and one-to-one guidance, the nurse teaches infants' families a variety of nursing skills, including basic neonatal nursing. After mastering these skills, the families can make sensory perception intervention on infants, which can not only improve the infants' excitatory-inhibitory function and enhance the brain regulatory effect but also raise their environmental adaptability, thus allowing infants to have better neuromotor and intellectual development [21]. Previous evidence found that the family participatory management mode can significantly increase the 18-month MDI and PDI scores of premature infants, with a similar effect on the growth and development of premature infants of different gestational ages [22].

The article "Effects of Family Participatory Nursing on Clinical Outcomes of Premature Infants in NICU and Families' Psychological Status" was published in 2022. Journal: Contrast Media Mol Imaging.

The families of premature infants often have unhealthy emotions such as anxiety and depression due to mother-baby separation and worry about the future development of premature infants. As reported [23], the adverse psychological status of the families of premature infants will reduce their compliance with the doctor's advice after discharge, harming the growth and development of premature infants. The psychological status of the families of premature infants is a concern in clinic, but further research is needed to clarify whether family participatory nursing can improve their psychological status. In this study, the families' somatization, depression, and anxiety factor scores and total score of SCL-90 in observation group were lower than those in control group, indicating that family participatory nursing can greatly improve the psychological status of the families of premature infants. A previous report showed that the families of premature infants in the NICU are generally in a nervous and anxious state, which will become worse due to their worry about the prognosis of premature infants and the fear of the isolated NICU environment, while family participatory nursing can effectively make parents less nervous and anxious [24]. With the emphasis on the importance of family participation, family participatory nursing allows the families to spend more time interacting with the infants, which greatly relieves their depression and anxiety [25]. Through cooperation and communication with the nurse during the nursing period, the families can have a better understanding of the conditions of infants and build up confidence. In addition, with the family participatory nursing mode, the potential of the families in the nursing intervention can be released and the workload of nurses can be reduced so that the nurse can spend more time on health education and skill training, thus benefitting the nursing work. In this study, each dimension score and total score of MPOC-20 in observation group were higher than those in control group. It can be seen that family participatory nursing can significantly raise the nursing satisfaction of the families of premature infants in the NICU because the families are taught scientific and effective nursing skills step by step, and parenting knowledge guidance is given throughout the nursing process in the family participatory nursing mode. This study is a single-center study with a small sample size and is not a randomized clinical study, the results of the study have some limitations and need to be confirmed in further multicentre randomized studies.

The article "Effects of Family Participatory Nursing on Clinical Outcomes of Premature Infants in NICU and Families' Psychological Status" was published in 2022. Journal: Contrast Media Mol Imaging.

## 5. Conclusion

In conclusion, family participatory nursing is of great significance in ameliorating the clinical outcomes of premature infants in the NICU, which can shorten the length of stay, improve feeding conditions, facilitate infant growth and development, and enhance their families' psychological status and nursing satisfaction.

## Figures and Tables

**Table 1:** Comparison of general clinical data between the two groups [*n* (%), *x̅* ± *s*].

Item		Observation group (*n* = 72)	Control (*n* = 78)	*t*/*χ*^2^ value	*P*-value
Sex	Male	40 (55.56)	41 (52.56)	0.135	0.713
	Female	32 (44.44)	37 (47.44)		

Gestational age (weeks)		31.17 ± 2.38	30.92 ± 2.06	0.689	0.492
Birth weight (kg)		1.38 ± 0.26	1.40 ± 0.31	0.4296	0.671
Apgar score (points)	1 min	7.89 ± 1.64	7.95 ± 1.59	0.227	0.820
	5 min	8.91 ± 1.63	8.94 ± 1.52	0.116	0.907

Mode of delivery	Transvaginal	46 (63.89)	45 (57.69)	0.602	0.438
	Cesarean section	26 (36.11)	33 (42.31)		
Maternal age (years)		30.13 ± 4.97	28.85 ± 5.06	1.561	0.121
Father's education level	Junior high school and below	3 (4.17)	5 (6.41)		0.826 ^*∗*^
	High school/secondary school	27 (37.50)	30 (38.46)		
	College degree or above	42 (58.33)	43 (55.13)		

Maternal education level	Junior high school and below	3 (4.17)	5 (6.41)		0.480 ^*∗*^
	High school/secondary school	25 (34.72)	33 (42.31)		
	College degree or above	44 (61.11)	40 (51.28)		

Participating family	Father	5 (6.94)	6 (7.69)	0.031	0.861
	Mother	67 (93.06)	72 (92.31)		

Note: *∗*Fisher's exact probability test.

**Table 2:** Comparison of hospitalization between the two groups [*n* (%), *x̅* ± *s*].

Group	Number of subjects	Hospital stay (d)	Oxygen therapy time (d)	Weight gain rate (g/d)	Nosocomial infection
Observation group	72	23.87 ± 3.64	12.76 ± 2.73	19.86 ± 4.53	6 (8.33)
Control group	78	27.03 ± 4.18	15.49 ± 3.42	18.05 ± 3.51	16 (20.51)
t/*χ*^2^-value		4.917	5.374	2.441	4.438
*P*-value		<0.001	<0.001	0.016	0.035

The article "Effects of Family Participatory Nursing on Clinical Outcomes of Premature Infants in NICU and Families' Psychological Status" was published in 2022. Journal: Contrast Media Mol Imaging.

**Table 3:** Comparison of feeding between the two groups [*n* (%), Fig. *x̅* ± *s*].

Group	Number of subjects	Time to full gastrointestinal feeding (d)	Daily milk intake (mL)	Exclusive breastfeeding	Feeding intolerance
Observation group	72	16.41 ± 3.64	79.25 ± 8.62	61 (84.72)	3 (4.17)
Control group	78	19.27 ± 4.02	63.49 ± 7.83	54 (69.23)	11 (14.10)
t/*χ*^2^ value		4.554	11.734	5.023	4.368
*P*-value		<0.001	<0.001	0.025	0.037

**Table 4:** Comparison of clinical outcomes between the two groups [*n* (%), *x̅* ± *s*].

Group	Number of subjects	Discharge weight (g)	Discharge weight *Z*-value	NBNA score (points) after 7 days of hospitalization	BSID score at 15 months of age (points)	
					MDI	PDI
Observation group	72	2.19 ± 0.24	1.245 ± 0.952	37.31 ± 3.89	96.47 ± 9.28	88.61 ± 9.92
Control group	78	2.07 ± 0.33	1.617 ± 0.916	35.63 ± 2.76	90.17 ± 8.53	81.43 ± 9.68
*t*-value		2.529	2.422	3.069	4.332	4.485
*P*-value		0.013	0.017	0.003	<0.001	<0.001

Note: NBNA is Neonatal Behavioral Neurometry Scale, BSID is Bailey Infant Development Scale, MDI is Mental Development Index, and PDI is Psychomotor Development Index.

**Table 5:** Comparison of SCL-90 scores between the two groups of children's families (*x̅* ± *s* (points).

Group	Number of subjects	Somatization	Forced	Interpersonal relationship	Depression	Anxious	Number of subjects	Hostility	Phobia	Paranoia	Psychotic	Total score
Observation group	72	1.32 ± 0.33	1.62 ± 0.46	1.57 ± 0.52	1.55 ± 0.40	1.68 ± 0.38	72	1.41 ± 0.42	1.22 ± 0.38	1.40 ± 0.43	1.27 ± 0.36	124.54 ± 19.67
Control group	78	1.47 ± 0.49	1.69 ± 0.59	1.69 ± 0.53	1.84 ± 0.61	1.97 ± 0.62	78	1.46 ± 0.49	1.27 ± 0.35	1.43 ± 0.41	1.29 ± 0.42	132.47 ± 22.56
*t*-value		2.181	0.806	1.398	3.413	3.420		0.668	0.839	0.437	0.312	2.286
*P*-value		0.031	0.422	0.164	0.001	0.001		0.505	0.403	0.663	0.756	0.024

**Table 6:** Comparison of MPOC-20 scores between the two groups of children's families (*x̅* ± *s* (points).

Group	Number of subjects	Authorization and cooperation	Provide basic information	Provide special information related to children	Coordination and overall care	Respect and supportive care	Total score
Observation group	72	5.42 ± 0.71	5.53 ± 0.93	5.57 ± 0.94	5.53 ± 0.82	5.31 ± 0.79	27.36 ± 2.26
Control group	78	4.83 ± 0.97	4.79 ± 0.88	4.96 ± 0.98	4.97 ± 0.85	4.87 ± 0.86	24.42 ± 2.37
*t*-value		4.221	5.007	3.884	4.100	3.255	7.761
*P*-value		<0.001	<0.001	<0.001	<0.001	0.001	<0.001

## Data Availability

The datasets used and analyzed during the current study are available from the corresponding author on reasonable request.
